The article "Downregulation of LINC01857 Increases Sensitivity of Gastric Carcinoma Cells to Cisplatin" was retracted in 2023. Reasons: unreliable results or conclusions; lack of ethics approval or compliance; concerns about the data; concerns about the results or conclusions.

# Downregulation of LINC01857 Increases Sensitivity of Gastric Carcinoma Cells to Cisplatin

**DOI:** 10.1155/2022/3325686

**Published:** 2022-05-11

**Authors:** Yun Chen, Yanli Wu

**Affiliations:** Pharmacy, Shulan (Hangzhou) Hospital Affiliated to Zhejiang Shuren University Shulan International Medical College, Hangzhou, Zhejiang 310004, China

## Abstract

**Background:**

The critical roles of long noncoding RNAs (lncRNAs) in the carcinogenesis and progression of cancers have been well documented. It was reported that lncRNAs were involved in chemotherapy resistance in various cancers. This study was aimed at clarifying the role of LINC01857 in cisplatin (DDP) resistance in gastric carcinoma (GC).

**Methods:**

The Cancer Genome Atlas (TCGA) database was used to analyze the expression of LINC01857 in GC tissues and normal tissues. The expression of LINC01857 in GC cells and DDP-resistant GC cells was detected by qRT-PCR. Cell viability and IC50 value were evaluated using the MTT assay. Moreover, cell apoptosis, migration, and invasion were determined using flow cytometry and Transwell assays, respectively. The expression of apoptosis-related proteins was examined by western blot.

**Results:**

TCGA database analysis revealed that LINC01857 expression was elevated in GC tissues compared with the normal tissues. qRT-PCR showed that the expression of LINC01857 was significantly higher in DDP-resistant cells than in GC and normal gastric cells. Knockdown of LINC01857 reduced cell viability in DDP-resistant cells. Moreover, LINC01857 downregulation promoted cell apoptosis and inhibited cell migration and invasion in DDP-resistant GC cells.

**Conclusions:**

LINC01857 was highly expressed in GC. Additionally, LINC01857 knockdown could facilitate the sensitivity to DDP and apoptosis and repressed cell migration and invasion in DDP-resistant GC cells, which provided a novel therapeutic target for chemotherapy resistance of GC in clinical practice.

## 1. Introduction

The incidence of digestive tract tumors was increasing annually due to the continuous growth of living standards and the formation of unhealthy eating habits [1]. Gastric carcinoma (GC), as the most common malignancy of the digestive system, is the third leading cause of cancer-related deaths in the eastern region [2]. GC has high morbidity and mortality rates with over 1 million new patients and approximately 760,000 GC-associated deaths each year, seriously threatening the life of people [3]. Generally, most GC patients were diagnosed at the advanced stage due to the nonspecific symptoms in the early stage of GC, resulting in that this disease was often not diagnosed or ignored [4, 5]. Despite advances in treatment over the past few decades, the prognosis for the patients with GC remains poor, with a 5-year survival rate of less than 25% [6, 7]. Cisplatin (DDP) is one of the effective chemotherapeutic agents and well known in first-line cancer treatment for various cancers, including GC [8]. However, the developed therapeutic resistance to DDP caused the common relapse and metastasis in GC patients [9]. Therefore, elucidating the detailed mechanism of DDP resistance in GC is imperative for discovering effective therapeutic targets of GC patients.

Long noncoding RNAs (lncRNAs) with over 200 nucleotides were considered transcriptional “noise” without any biological function and the ability to encode proteins [10–12]. Recent studies found that lncRNAs presented aberrant expression in several types of tumors and participated in the growth, metastasis, invasion, and apoptosis of tumor cells via different signaling pathways [13]. It was reported that promoting tumor cell apoptosis has always been the main therapeutic direction for tumor treatment in clinic [14]. Accumulating evidence indicated that lncRNAs could regulate drug resistance and apoptosis of tumor cells via interacting with the key apoptosis regulators [15–17]. LINC01857, a newly discovered lncRNA located on human chromosome 2q33.3 [18], was found to be highly expressed in a wide variety of human cancers. For example, LINC01857 was significantly upregulated in breast cancer and involved in its progression by modulating the activation of CREB1 via interacting with CREBBP [19]. LINC01857 promoted cell growth, migration, and invasion via modulating the miR-1281/TRIM65 axis in glioma and was also proven to be increased in liver cancer [20, 21]. Additionally, LINC01857 facilitated gastric carcinogenesis by targeting miR-200b [22]. Nonetheless, the role of LINC01857 in DDP resistance in GC remains elusive.

Herein, this study mainly investigated the function of LINC01857 in DDP resistance of GC, aimed at providing evidence for GC clinical treatment.

## 2. Methods and Materials

### 2.1. Database Analysis and Clinical Data Collection

The GC gene expression profiles (mRNAs, standardized RNAseqV2 RSEM) of 30 normal gastric specimens and 343 GC specimens were collected from the Cancer Genome Atlas (TCGA) database.

### 2.2. Cell Culture and Transfection

The human gastric epithelial cell line (GES-1 cells), human GC cell lines (BGC823 and SGC7901 cells), and human DDP-resistant GC cell lines (BGC823/DDP and SGC7901/DDP cells) were provided by the American Type Culture Collection (ATCC; Manassas, Virginia, USA). The above-mentioned cell lines were cultured in PRMI-1640 medium containing 10% FBS (Invitrogen, Carlsbad, CA, US) at 37°C with 5% CO_2_. Small interfering RNAs (siRNAs) against LINC01857 (si-LINC01857#1: 5′-ATCTAACAGTTTCCGCTATTTTG-3′, si-LINC01857#2: 5′-AAGAGATAGAGGAAAAATGGATT-3′, and si-LINC01857#3: 5′-AGGAAAAATGGATTCAACAAATG-3′) and the negative control (si-NC) were provided by GenePharma (Shanghai, China). Cell transfection was performed using Lipofectamine 2000 (Invitrogen, Carlsbad, CA, USA).

### 2.3. qRT-PCR

Total RNA was isolated using Trizol reagents (Invitrogen). Then, the RNA (100 ng per sample) was reverse-transcribed into cDNA synthesis using a PrimeScript RT kit (TaKaRa, Tokyo, Japan). Subsequently, PCR amplification was carried out with the ABI7500 and SYBR Green qRT-PCR kit to detect the relative expression of LINC01857. The reaction system include the following: 1 *μ*L cDNA template, 7.8 *μ*L ddH20, 10 *μ*L SYBR Premix EX Tap (ZX), 0.4 *μ*L each of upstream and downstream primers, and 0.4 *μ*L ROX reference dye II (50x). Reaction conditions (40 cycles) were as follows: predenaturation: 95°C, 30 s; denaturation: 95°C, 5 s; annealing: 60°C, 34 s; and extension: 95°C, 15 s. Each sample was repeatedly tested 3 times. GAPDH served as an internal reference, and the data were analyzed by the 2^−ΔΔCt^ method [23]. All operations were conducted in strict accordance with the corresponding instructions. Primer sequences are presented in Table 1.

### 2.4. DDP Sensitivity Test

3-(4,5-Dimethyl-2-thiazolyl)-2,5-diphenyl-2H-tetrazolium bromide (MTT; Sigma-Aldrich) was used to detect the viability of GC or DDP-resistant GC cells under various DDP concentrations to determine and visualize the semi-inhibitory concentration (IC50) value of DDP. IC50 values were defined as DDP concentrations corresponding to 50% of cell viability inhibition rates in the curve.

### 2.5. Transwell Assay

Transwell assays were used to detect the invasion and migration ability of the cells. The transfected cells were collected. The cell density was adjusted to 4 × 10^4^ and suspended in a serum-free medium containing 1 *μ*g/mL mitomycin C. Then, the cells were inoculated in the upper chamber precoated with Matrigel, and 10% bovine fetal serum was added to the lower chamber. After 24 h of incubation at 37°C, the substrate and cells in the upper chamber that had not passed through the membrane surface were wiped off. Then, the cells were washed and fixed with paraformaldehyde for 10 min. Subsequently, the cells were stained with 0.5% crystal violet. Cell invasion was observed with a microscope. The cell migration assay was similar to the invasion assay, except that Matrigel was not added to the upper chamber of the Transwell.

### 2.6. Flow Cytometry

The transfected BGC823/DDP and SGC7901/DDP cells were collected and dyed with Annexin V-FITC (3 *μ*L) and propidium iodide (5 *μ*L) at room temperature for 15 min in the dark. Finally, each sample was immersed in 1× binding buffer (300 *μ*L) for apoptosis analysis using the FACSCalibur system (BD Biosciences, US).

### 2.7. Western Blot

Total proteins were extracted using the RIPA buffer, and cell protein concentration was determined by the bicinchoninic acid (BCA) kit (Pierce, Rockford). Then, the protein samples with equal amount were separated on 10% SDS-PAGE before transferring them to the PVDF membranes. After a 2 h blocking with 5% defatted milk at 37°C, the membranes were incubated overnight in TBST buffer diluted with the primary antibodies cle-caspase-3 (Abcam, Cambridge, MA, USA, ab32042, 1 : 1000), Bax (Abcam, ab32503, 1 : 1000), Bcl-2 (Abcam, ab32124, 1 : 1000), and GAPDH (Abcam, ab8245, 1 : 1000) at 4°C and then incubated with the horseradish peroxidase- (HRP-) conjugated secondary antibody at 70°C for 2 h. GAPDH was used as the internal reference. The protein band images were analyzed by a Tanon detection system after development with enhanced chemiluminescence (ECL) reagents (Thermo, US), and the antigen-antibody response was observed by ECL.

### 2.8. Statistical Analysis

All data were analyzed using GraphPad Prism 8. Experimental data were expressed as the mean ± standard deviation (SD) and compared using one-way analysis of variance (ANOVA) and Student's *t*-test. Differences with *P* value < 0.05 were deemed significant. The experiment was repeated 3 times.

## 3. Results

### 3.1. LINC01857 Was Highly Expressed in GC Tissues and Cells

To determine LINC01857 expression in GC, we analyzed its expression profile in GC through TCGA database. The data suggested that LINC01857 was evidently elevated in GC tissues in comparison to normal tissues (Figure 1(a)). Moreover, higher expression of LINC01857 was observed in GC cells compared with GES-1 cells. Further analysis revealed that the expression of LINC01857 was significantly upregulated in DDP-resistant GC cells relative to GC cells (Figures 1(b) and 1(c)).

### 3.2. DDP Sensitivity Was Decreased in DDP-Resistant GC Cells

In order to investigate the role of LINC01857 in DDP-resistant GC cells, we determined the IC50s of BGC823 and SGC7901 (parent cells), as well as DDP-resistant GC cells (BGC823/DDP and SGC7901/DDP cells). The MTT assay identified that the IC50 value was higher in SGC7901/DDP cells than in BGC823 and SGC7901 cells (Figures 2(a) and 2(b)).

### 3.3. LINC01857 Expression Was Decreased in DDP-Resistant GC Cells Transfected with si-LINC01857#3

To clarify the role of LINC01857 in DDP-resistant GC cells, si-LINC01857#1, si-LINC01857#2, and si-LINC01857#3 were transfected into DDP-resistant GC cells. Through qRT-PCR analysis, we found that the inhibition of si-LINC01857#3 was the most significant in BGC823/DDP cells (Figure 3(a)). Thus, si-LINC01857#3 was selected for the next experiments. qRT-PCR detection identified that the expression of LINC01857 was significantly reduced in BGC823/DDP and SGC7901/DDP cells transfected with si-LINC01857#3 (Figure 3(b)).

### 3.4. LINC01857 Knockdown Elevated DDP-Resistant GC Cell Sensitivity to DDP

As shown in Figures 4(a) and 4(b), we found that downregulation of LINC01857 effectively enhanced the sensitivity of BGC823/DDP and SGC7901/DDP cells to DDP. In addition, si-LINC10857#3 transfection induced the apoptosis of DDP-resistant GC cells (Figure 5(a)). Furthermore, the results in western blot demonstrated that decrease in LINC01857 promoted the expression of cle-caspase-3 and Bax and inhibited the expression of Bcl-2 in BGC823/DDP and SGC7901/DDP cells, suggesting that LINC01857 could modulate the expression of apoptosis-related proteins (Figure 5(b)). Moreover, Transwell assays showed that the invasion and migration abilities of DDP-resistant GC cells were inhibited after transfection with si-LINC10857#3 (Figures 6(a) and 6(b)).

## 4. Discussion

Drug resistance commonly caused the treatment failure of advanced GC patients and is a hurdle that needs effective solutions. The clinical practice guidelines recommend platinum for the postoperative chemotherapy in GC patients at an advanced stage [24]. There are still a large number of GC patients who benefit little from postoperative chemotherapy due to chemical resistance [25]. In fact, in addition to surgical resection, chemotherapy is the main method for the treatment of GC patients with GC, which can significantly reduce the incidence of postoperative recurrence and metastasis [26]. However, chemotherapy resistance during postoperative treatment significantly limits its clinical application. Thus, it is urgent to investigate the underlying mechanism of drug resistance in GC treatment. In this study, our data demonstrated that LINC01857 was elevated in GC patients and significantly higher in DDP-resistant GC cells compared with their parents. Functional assays indicated that knocking down LINC01857 led to lower IC50s of DDP-resistant GC cells and enhanced apoptosis, suggesting that LINC01857 might be a potential therapeutic strategy for drug resistance of GC.

The critical roles of lncRNAs in tumor drug resistance have been well documented [27–29]. For example, the study by Zhu et al. found that MT1JP inhibited the tumorigenesis of breast cancer and enhanced DDP sensitivity in breast cancer cells through competitive binding with miR-24-3p [30]. Another research suggested that downregulation of CASC2 promoted DDP resistance in GC by stimulating miR-19a [31]. As a newly discovered lncRNA, LINC01857 has been relatively rarely studied in GC. According to TCGA database, we found that LINC01857 was highly expressed in GC patients, which was similar to the research conducted by Chen et al. [22]. High expression of LINC01857 was also found in DDP-resistant GC cells, suggesting that LINC01857 might be closely associated with DDP resistance in GC.

In GC, the detailed mechanism of LINC01857 in DDP sensitivity was still uncertain. To study the underlying mechanism of LINC01857 in DPP resistance in GC, we knocked down LINC01857 in DDP-resistant GC cells. The results showed that LINC01857 knockdown caused the reduced IC50s and notably enhanced DDP-resistant GC cell apoptosis. Apoptosis-related proteins, as indicators reflecting apoptosis, could be used as direct evidence of apoptosis through detection of their expression levels [32]. As a classic proapoptotic factor in the Bcl-2 family, Bax expression was lowly expressed in cells but dramatically increased in the apoptotic cells [33, 34]. Caspase-3 belongs to the caspase family and played a vital role in the execution of apoptosis [35, 36]. In this research, significantly reduced Bcl-2 and obviously elevated cle-caspase-3 and Bax protein expression levels were observed after knockdown of LINC01857, indicating that LINC01857 could increase the sensitivity of DDP-resistant GC cells. Moreover, our data showed that LINC01857 knockdown significantly repressed cell migration and invasion in DDP-resistant GC cells.

In this research, we explored the role of LINC01857 in DDP-resistant GC cells. However, this study still has some limitations of improvement. We did not detect LINC01857 expression in GC patients with or without failed chemotherapy. Moreover, multiple studies suggested that lncRNAs could alter downstream target gene expression by modulating miRNAs; thus, the in-depth study on the downstream genes of LINC01857 is required. In addition, *in vivo* experiments are warranted for further exploration. We will carry out more experiments in the future to improve our research.

To sum up, our findings revealed that LINC01857 downregulation facilitated cell apoptosis, inhibited cell migration and invasion, and increased the sensitivity of DDP-resistant GC cells to DDP, providing a potential target of DDP resistance in GC.

## Figures and Tables

**Figure 1:** LINC01857 was highly expressed in GC tissues and cells. (a) LINC01857 expression in GC tissues was evaluated using TCGA database. (b) LINC01857 expression in GES-1, BGC823, and BGC823/DDP cells was measured by qRT-PCR. (c) LINC01857 expression in GES-1, SGC7901, and SGC7901/DDP cells was detected by qRT-PCR. ^∗∗^*P* < 0.01, ^∗∗∗^*P* < 0.001.

**Figure 2:** DDP sensitivity was decreased in DDP-resistant GC cells. (a) IC50s of BGC823 and BGC823/DDP cells were measured by the MTT assay. (b) IC50s of SGC7901 and SGC7901/DDP cells were detected by the MTT assay. ^∗^*P* < 0.05.

**Figure 3:** LINC01857 expression was decreased in DDP-resistant GC cells transfected with si-LINC01857#3. (a) LINC01857 expression in BGC823/DDP transfected with si-LINC01857#1, si-LINC01857#2, and si-LINC01857#3 was detected by qRT-PCR. (b) LINC01857 expression in BGC823/DDP and SGC7901/DDP cells transfected with si-LINC01857#3 by qRT-PCR. ^∗^*P* < 0.05, ^∗∗^*P* < 0.01.

**Figure 4:** LINC01857 knockdown elevated DDP-resistant GC cell sensitivity to DDP. (a) Changes of IC50 in BGC823/DDP cells transfected with si-LINC01857#3 were evaluated by the MTT assay. (b) Changes of IC50 in SGC7901/DDP cells transfected with si-LINC01857#3 were determined by the MTT assay. ^∗^*P* < 0.05.

**Figure 5:** Downregulation of LINC01857 enhanced the apoptosis of DDP-resistant GC cells. (a) Cell apoptosis was assessed by flow cytometry. (b) Changes of apoptosis-related proteins in BGC823/DDP and SGC7901/DDP cells transfected with si-LINC01857#3 were determined by western blot. ^∗^*P* < 0.05; ^∗∗^*P* < 0.01.

**Figure 6:** Downregulation of LINC01857 inhibited the invasion and migration of DDP-resistant GC cells. (a) Transwell invasion assay was used to detect cell invasion in DDP-resistant GC cells transfected with si-LINC01857#3 or si-NC. (b) Transwell migration assay was used to detect cell migration in DDP-resistant GC cells transfected with si-LINC01857#3 or si-NC. ^∗∗^*P* < 0.01.

**Table 1:** Primer sequences.

Gene	Forward (5′-3′)	Reverse (5′-3′)
LINC01857	CAGGACTCCATTAAGGACTC	AACATCGATGTGTCCCAGGA
GAPDH	CGCTCTCTGCTCCTCCTGTTC	ATCCGTTGACTCCGACCTTCAC

## Data Availability

The labeled dataset used to support the findings of this study is available from the corresponding author upon request.
